# An Improved CNN Architecture to Diagnose Skin Cancer in Dermoscopic Images Based on Wildebeest Herd Optimization Algorithm

**DOI:** 10.1155/2021/7567870

**Published:** 2021-08-27

**Authors:** Biying Zhou, Behdad Arandian

**Affiliations:** ^1^School of Computer, Weinan Normal University, Weinan 714099, Shaanxi, China; ^2^Department of Electrical Engineering, Dolatabad Branch, Islamic Azad University, Isfahan, Iran

## Abstract

Skin cancer is one of the most common types of cancers that is sometimes difficult for doctors and experts to diagnose. The noninvasive dermatoscopic method is a popular method for observing and diagnosing skin cancer. Because this method is based on ocular inference, the skin cancer diagnosis by the dermatologists is difficult, especially in the early stages of the disease. Artificial intelligence is a proper complementary tool that can be used alongside the experts to increase the accuracy of the diagnosis. In the present study, a new computer-aided method has been introduced for the diagnosis of the skin cancer. The method is designed based on combination of deep learning and a newly introduced metaheuristic algorithm, namely, Wildebeest Herd Optimization (WHO) Algorithm. The method uses an Inception convolutional neural network for the initial features' extraction. Afterward, the WHO algorithm has been employed for selecting the useful features to decrease the analysis time complexity. The method is then performed to an ISIC-2008 skin cancer dataset. Final results of the feature selection based on the proposed WHO are compared with three other algorithms, and the results have indicated good results for the system. Finally, the total diagnosis system has been compared with five other methods to indicate its effectiveness against the studied methods. Final results showed that the proposed method has the best results than the comparative methods.

## 1. Introduction

Skin cancer is the most common malignant cancer of the body [1]. This cancer is caused by the uncontrolled and abnormal growth of skin cells. Ultraviolet rays from sunlight and tanning lamps cause genetic changes in the nucleus of skin cells [2]. If the body's immune system fails to repair the damage, skin cells begin to grow rapidly and unrestrained, initially appearing as fast-growing moles with bleeding, tumors, or wounds that do not heal such that if not treated, it spread to other areas (metastasis) [3].

One of the most dangerous types of skin cancer is melanoma. Melanoma is the deadliest type of skin cancer. Melanoma commonly begins with changes in an old or normal mole or suddenly appears as a black or dark brown area on the skin. Early detection is very important [4]. Here are the important points in early diagnosis. There is usually no symmetry in the skin lesion, and one half of the lesion is different from the other. The margin of the lesion is not clear and is not well diagnosable from the surrounding healthy skin. The lesion may be seen in several different colors. Brown and black are more common, and red, white, and blue are less common [5]. The diameter of the lesions is usually more than six millimeters. The last important symptom is the difference between a fleshy spot or a brown spot and other spots on the body, which usually begin to change shape and color or cause itching and bleeding [6].

Melanoma, as one of the skin cancers, is responsible for 50% of deaths associated with skin cancers. The source of this disease is in the epidermal and dermal layers of the skin [7]. This disease is formed by the accumulation of melanin granules, and it is spread to the outermost layer of the skin. Since determining the extent of the lesion and somehow extracting the exact boundary between the lesion and the background is one of the most influential parameters in clinical methods of diagnosing cancerous lesion, therefore, providing lesion diagnosis methods is of great importance [8].

Goldman first invented the dermatoscope, which evaluates changes in skin pigmentation under disease conditions. Dermatologists then used this device as a suitable and noninvasive tool to observe skin lesions. With the development of science in recent years, the digital dermatoscope has been replaced by conventional dermatoscopes with the ability to capture and store skin images. Therefore, it is possible to provide commercial software packages to help diagnose some skin lesions, create databases, and create a medical resume for each patient [9].

Melanoma diagnosis by modern smart devices, in the early stages of its formation, is a very important issue that has involved many researchers [10]. Meanwhile, melanoma due to its high prevalence has attracted a large amount of research. For example, Razmjooy et al. presented a new well-organized technique to diagnose the melanoma from dermoscopy images. Firstly, the additional scales were removed using edge detection and smoothing. Then, the data were segmented, and mathematical morphology was used as postprocessing section. They also used an optimized multilayer perceptron (MLP) for the final classification. The optimization was based on the World Cup Optimization (WCO) Algorithm. Simulation results indicated the high accuracy of the system based on the authors explanations [11].

Pathan et al. proposed an automatic system for the diagnosis of the melanoma. The method contained a set of sequential stages. 2D Gabor filters were used for detection of the pigment network masks. A machine learning based on the rules was then produced from the pigment network masks to detection of the typical and atypical pigment network patterns. The method was implemented on PH2 dataset. The method was also compared with some state-of-the-art techniques from the literature to show the method effectiveness [12].

Xu et al. presented another automatic CAD-based technique for early diagnosis of melanoma. In the method, the noise of the input images was first reduced by a median filter. Then, a new optimized method for segmentation of the region of interest was proposed based on the convolutional neural network (CNN). To improve the CNN efficiency, it is optimized based on the satin bowerbird optimization (SBO) algorithm. Afterward, the main features of the region of interest were extracted for the next step. Because of the large volume of the features, an optimized feature selection based on the SBO algorithm was also utilized. At last, the images were classified based on a support vector machine (SVM). Final results were implemented on the American Cancer Society database, and the results were compared with some state-of-the-art methods to show the method dominance [13].

As can be observed from the literature, several and different techniques were proposed for skin cancer diagnosis. However, providing an optimal technique for the diagnosis system is not too simple, and each of them has its advantages and shortages. Moreover, using deep learning for this purpose is also too useful. However, using the combination of these works is not provided or may be too rare. Therefore, in this paper, a new diagnosis method was proposed for melanoma detection. The method extracted features of the images by the help of a CNN that is done from the melanoma dermoscopic images. Afterward, the Water Strider Algorithm (WSA) is for optimal selection of the only relevant features. Here, we utilized WSA as a feature selector from deep features which are generated by the CNN with large redundancy. The results showed that this process can develop the diagnosis accuracy of the melanoma. The next sections of this paper are organized as follows. In Section 2, the main materials and methods are explained. This section contains the structure of the CNN and how the CNN can be used for the features extraction.  Section 3 describes about the definition of the Wildebeest Herd Optimization Algorithm. In Section 4, the utilized dataset has been described.  Section 5 includes the simulation results and the discussions about the results. The paper has been concluded in Section 6.

## 2. The Convolutional Neural Network

### 2.1. CNN-Based Features Extraction

The present paper uses a convolutional neural network (CNN) for establishing the feature extraction of the melanoma dermoscopic images. A pretrained model of CNN has been trained on the dataset that includes several of images on different classes. So, the transfer learning has been implemented by transferring weights which were already trained and reserved into the structure of the pretrained model, like Inception, in this paper. Three main parameters are considered for the CNN: Filter size, Stride, and Max pooling. The present study uses size 2 filters, and also size 2 stride parameter and 2 × 2 Max pooling filter are employed. The main target of convolutional layers here is to provide a proper features extraction from the input images. Here, we used different convolutional layers that have been implemented to extract various features like texture, edges, high-lighted patterns, and colors from the images.

Three fully connected layers are then used for classification. We also used Softmax as activation function to provide a binary output (positive melanoma and negative melanoma). The last concatenation layer that includes the extracted features has been kept, and the top layers such as the Flatten, Drop out, and the Dense layers which the later performs classification have been removed. The weights have been updated by RMSprop optimizer, and cross entropy loss function and learning rate are set as 1*e* − 4. The input shape for the feature extractor (Inception) is [225, 225, 3].  Figure 1 shows an overview of Inception network [14].

A significant disadvantage of the pretrained models like Inception is that their construction needs a big memory as well as storage capacity, that makes a high time complexity for the system. Therefore, some statistical operations are added to ignore immaterial features. In the following, these features have been briefly given [14].

#### 2.1.1. Tree-Based Classifier

This feature is one of the most popular methods to advance the classification ratio. In addition to high accuracy, they are simple and robust. For all decision trees, node importance has been evaluated by Gini importance, and this is given in the following formula:

(1) $$\begin{array}{c} n_{k}=w_{k}C_{k}-w_{k}^{\text{left}}C_{k}^{\text{left}}-w_{k}^{\text{right}}C_{k}^{\text{right}}, \end{array}$$

where *w*_*k*_ signifies the weighted number of samples that reaches the node *k*, *n*_*k*_ describes the importance of node *l*, *C*_*k*_ defines the contamination value of the *k*^th^ node, and left and right represent the child nodes from the left and the right splits on the *k*^th^ node, respectively. The importance of the features is then evaluated.

(2) $$\begin{array}{c} f_{i}=\frac{\sum_{j:\text{node }k\text{ splits on feature }i}n_{k}}{\sum_{j\in \text{all nodes}}n_{j}}, \end{array}$$

where *n*_*k*_ describes the importance of the *k*^th^ node and *f*_*i*_ describes the importance of feature *i*.

Normalize the values in the range [0, 1] by dividing the sum of all feature importance values, i.e.,

(3) $$\begin{array}{c} \bar{f_{i}}=\frac{f_{i}}{\sum_{k\in \text{all nodes}}f_{k}}. \end{array}$$

Finally, the sum of the importance value in the features for the trees is evaluated and then divided by the total number of trees, i.e.,

(4) $$\begin{array}{c} Rf_{i}=\frac{\sum_{k\in \text{all trees}}\bar{f_{i}}}{T}, \end{array}$$

where *Rf*_*i*_ describes the importance of the *i*^th^ feature that are evaluated from all trees, where $\bar{f_{i}}$ describes the normalized feature importance for the *i*^th^ feature in the *j*^th^ tree and *T* defines the total number of trees.

#### 2.1.2. Chi-Square

This feature has been implanted to eliminate the features with high correlation values by evaluating their dependency. This is evaluated on all classes between each feature:

(5) $$\begin{array}{c} \psi^{2}=\overset{n}{\underset{j=1}{\sum }}\frac{{\left(Y_{j}-E_{j}\right)}^{2}}{E_{j}}, \end{array}$$

where *Y*_*j*_ and *E*_*j*_ represent the real and the expected feature values, respectively.

Here, after establishing Chi-square, the feature vector has been minimized for the dataset.

## 3. Wildebeest Herd Optimization Algorithm

The main target of optimization is to provide the most desirable solution to the problem by considering its limitations and other features. Numerous solutions have been introduced for solving an optimization problem. Formerly, classical methods like Pontryagin maximum principle [15] and distributed newton method [16] were used for this purpose. However, by increasing the complexity of the problems, the classical methods have been weakened such that they failed in solving some kinds of NP-hard problems. This made the researchers to move toward and offer newer methods to resolve the classical optimization methods' issues. Metaheuristic algorithms are some kinds of new optimization algorithms that recently are used extensively for this purpose. In recent years, lots of different versions for metaheuristic algorithms have been introduced, for example, Manta-Ray Foraging Optimization (MRFO) [17], World Cup Optimization (WCO) Algorithm [18], Locust Swarm Optimization (LSO) Algorithm [19], and Wildebeest Herd Optimization (WHO) Algorithm [20].

In this study, the Wildebeest Herd Optimization (WHO) Algorithm [20] has been utilized for optimizing of our deep network. The main reason for selecting this algorithm is that it is too recent among different types of the metaheuristic algorithms. Also, its results on the benchmark functions based on the paper provide too better results. This makes us to use this metaheuristic technique to improve the efficiency of the proposed CNN. The WHO algorithm has been inspired from the behavior of food searching by the Wildebeests. Wildebeests are social mammal animals which travel to find food sources. The male sex challenges with other competitors to get females for mating.

The Wildebeest Herd Optimization (WHO) Algorithm starts by random initializing a number of population (wildebeests) as candidates. The population is limited between the lower (*X*_min_), and the higher (*X*_max_) boundaries, i.e.,

(6) $$\begin{array}{c} X_{i}\in \left[X_{\text{min}},\;X_{\text{max}}\right], \end{array}$$

where *i*=1,2,…, *N*.

The milling action is then used for local movement of the wildebeest individuals. The phase is modeled by considering a consistent number (*n*) as the minor random movement based on the solution spaces and continuing to find the optimal position. A random phase *Z*_*n*_ has been employed by the candidates in position *X* that should frequently search for the small random phase positions. A tunable length is accomplished by a random step size to the candidates. Consequently, the local experimental phase *Z*_*n*_ is obtained in the following formula:

(7) $$\begin{array}{c} Z_{n}=X_{i}+\varepsilon \times \theta \times \nu , \end{array}$$

where *ε* signifies the learning rate variable, *X*_*i*_ describes the candidate number *i*, *θ* represents a randomly uniform value ranged between 0 and 1, and *ν* defines a random unit vector.

Then, a constant number (*n*) of minor random candidates is evaluated, and the wildebeest updates its position to get an optimal random location, i.e.,

(8) $$\begin{array}{c} X_{i}=\alpha_{1}\times Z_{n}^{*}+\beta_{1}\times \left(X_{i}-Z_{n}^{*}\right), \end{array}$$

where *α*_1_ and *β*_1_ describe the leader variables to lead the local movement of the candidates.

The last phase is to model the swarm instinct of the wildebeests. This is simulated once the other candidates are positioned in a location with proper food source, i.e.,

(9) $$\begin{array}{c} X_{i}=\alpha_{2}\times X_{i}+\beta_{2}\times X_{h}, \end{array}$$

where *X*_*h*_ defines a random candidate and *α*_2_ and *β*_2_ represent the leader variables to lead the local movement of the crew.

In the Wildebeest Herd optimization algorithm, there is another term to avoid the candidates from moving to spaces with insufficient food source. This term is mathematically modeled as follows:

(10) $$\begin{array}{c} X_{i}≔X_{i}+\theta \times \left(X_{\max}-X_{\min}\right)\times \bar{v}, \end{array}$$

where $\bar{v}$ describes a random unit vector.

Another term in the algorithm is to simulate the crowded spaces. The crowd happens when there is a wide fertility for the grass. This term is named “individual pressure.” Based on this term, a challenge is accomplished and the strongest candidate demolishes the others using the following equation:

(11) $$\begin{array}{c} \text{if}\left(\left\|X^{*}-X_{i}\right\|\right)<\eta ,\;\left(\left\|X^{*}-X_{i}\right\|\right)>1\\ \text{then}:\;X_{i}=X^{*}+\varepsilon \times \hat{n}, \end{array}$$

where *η* signifies a threshold to avoid crowding in the spaces and $\hat{n}$ describes exploitable parts number close to the optimum solution point.

And the final phase is to simulate the swarm social memory to offer better positions that is called swarm social memory and is obtained by the following equation:

(12) $$\begin{array}{c} X=X^{*}+0.1\times \hat{\nu }. \end{array}$$

By combination of the concept of the Wildebeest Herd Optimization Algorithm with the Inception network, the total method of the proposed system has been determined as follows:

1. Extracting deep features from Inception.
2. Initializing solutions for the Wildebeest Herd. The Herd follows the leader during searching the fertile grass source (solution space).
3. Attempting the wildebeest to catch the best fertile food source based on exploration and exploitation terms in the algorithm.
4. All stages are repeated until the termination criteria have been reached.

## 4. The Database

The present study uses International Skin Imaging Collaboration (ISIC-2008) for validation. This archive defines an international attempt to progress the research studies for the melanoma diagnosis which is supported by the International Society for Digital Imaging of the Skin (ISDIS). This dataset includes the largest widely available collection of dermoscopic images for skin lesions. The dataset includes over 13,000 dermoscopic images that have been gathered from international clinical centers and collected from different devices within the centers. This international collaboration is to guarantee to collect a proper dataset. Also, a subset of the images has been labeled by the experts.  Figure 2 shows some examples of the ISIC-2008 dataset [21].

## 5. Simulation Results

Because the WHO algorithm is a metaheuristic and has stochastic nature, the achieved results of this algorithm may change during different executions. Consequently, in this study, the training method by the WHO algorithm has been repeated for 30 times and the best network has been used for the analysis. The WHO algorithms and the Inception network have been programmed in MATLAB 2019b 64 bit version and executed on computation environment of Intel Core i7Intel processor CPU 2.00 GHz, 2.5 GHz, and 32 GB RAM with and two SLI GeForce Titan GPUs and 64 bit operating system. The convolutional neural networks were under Google lab network.

The section confirms and discusses about the results of the proposed skin cancer diagnosis system. The method is performed to the ISIC-2008 dataset. For the dataset, the segmented cancer has been assessed by a comparative study with the expert's ground truth image.

To assess the efficiency of the suggested method, the average value of both best values and the worst values (Max) along with standard deviation (Std) and computational time has been evaluated. The mathematical definitions of all indicators are given as follows:

(13) $$\begin{array}{c} \text{ACC}=\frac{\left(\text{TP}+\text{TN}\right)}{\left(\text{FP}+\text{TP}+\text{TP}+\text{FN}\right)},\\ \text{SPC}=\frac{\text{TN}}{\text{FP}+\text{TN}},\\ \text{SNS}=\frac{\text{TP}}{\text{TP}+\text{FN}},\\ F_{\text{score}}=2\times \frac{\text{SPC}\times \text{SNS}}{\text{SPC}+\text{SNS}}, \end{array}$$

where TP is the true positive, TN is the true negative, FP is the false positive, and FN is the false negative, and ACC, SPC, and SNS represent the accuracy, specificity, and sensitivity, respectively.

And the optimization is based on the following equation:

(14) $$\begin{array}{c} {\text{Best}}_{\text{ACC}}=\text{Max ACC,}\\ {\text{fit}}_{\text{Best}}={\text{Min Fit}}_{i},\\ {\text{fit}}_{\text{worst}}={\text{Max Fit}}_{i},\\ {\text{fit}}_{\text{avg}}=\frac{1}{m}\overset{N}{\underset{i=1}{\sum }}{\text{Fit}}_{i},\\ \text{Std}=\sqrt{\frac{1}{m-1}\times \overset{m}{\underset{i=1}{\sum }}{\left({\text{Fit}}_{i}-{\text{fit}}_{\text{avg}}\right)}^{2}}\;,\\ i=1,2,\ldots ,m\text{,} \end{array}$$

where *m* describes the number of evaluations and Fit_*i*_ signifies the fitness function value.

Once Inception trains the skin cancer images continuously in the epochs, these rapid ups and downs are gradually minimized in the future training part.

After feature extraction based on Inception, the WHO algorithm has been performed to optimal selection of the features and to eliminate the useless features. Here, the results of the proposed WHO-Inception have been compared with some state-of-the-art optimization algorithms including Chimp optimization algorithm (ChOA) [22], Biogeography-Based Optimizer (BBO) [23], and Locust Swarm Optimization (LS) [24] for feature selection. The parameter setting of the utilized optimization algorithms is reported in Table 1.

Here, the feature selection methods have been employed for optimal selection of the generated feature vector from Inception to provide just the useful relevant features. Some of the parameters are selected similar to fair comparison. All of the algorithms have 15 iterations and 30 number of candidates. All of the algorithms are run for 35 independent runs to offer consistent results.  Table 2 reports the results of four measurement indicators applied by the before mentioned optimization algorithms of the feature selection for the dataset.

As can be observed from Table 2, the proposed WHO algorithm has the higher efficiency toward the other comparative algorithms in all four metrics followed by LS, ChOA, and BBO, respectively. The best results of fit_worst_ indicated that the proposed WHO algorithm provides the best value of the fitness function against the others. Also, LS is placed on the second rank.  Figure 3 shows the running time of the analyzed algorithms.

As can be observed from Figure 3, the proposed WHO algorithm considers the fastest results among all of the compared algorithms followed by ChOA and BBO, respectively, while LS has the slowest results.  Figure 4 shows the simulation results for number of selected features based on the studied comparative algorithms.

As can be observed from Figure 4, the proposed WHO algorithm with 210 features provided less features than other algorithms. BBO and LS are placed in the second and the third ranks with 314 and 352 selected features, respectively. The largest features have been selected by ChOA.

In the following part, the image similarity and statistical measures like dice coefficient (DC), accuracy (ACC), specificity (SPC), PPV, NPV, and sensitivity (SNS) are evaluated. The mathematical model of the parameters is given as follows:

(15) $$\begin{array}{c} \text{Ds}=\frac{2\times \text{TP}}{\left(\left(\text{FP}+\text{TP}\right)+\left(\text{TP}+\text{FN}\right)\right)},\\ \text{PPV}=\frac{\text{TP}}{\text{TP}+\text{FP}},\\ \text{NPV}=\frac{\text{TN}}{\text{TN}+\text{FN}}, \end{array}$$

where TP is the true positive, TN is the true negative, FP is the false positive, and FN is the false negative.

The final results are compared with 5 state-of-the-art methods from the literature including Dorj's [25], Linsangan's [26], Thanh's [6], Khan's [2], and Angurana's [27].  Table 3 reports the simulation results of the suggested method compared with other state-of-the-art methods.

Figure 5 shows the bar plot of the classification rate. It can be observed from the results that the presented methodology offers the highest accuracy compared with the other methods from the literature.

As can be observed from Table 1, the suggested technique with 96% accuracy offers the uppermost efficiency among the other comparative methodologies. Similarly, Dorj's method and Angurana's method with 91% have the second rank in the comparison. Likewise, Linsangan's, Khan's, and Thanh's methods with 89%, 88%, and 87%, respectively, are in the next ranks. Also, the suggested method with 96% sensitivity as the highest value against the others indicates the method's higher consistency than the others. Furthermore, higher value of PPV and NPV for the suggested method against the others designates its higher condition occurrence for handling the likelihood of a test identifying the cancer. In addition, higher results for the specificity of the suggested technique indicate its sophisticated occurrence-independent achievement.

## 6. Conclusions

Skin cancers are one of the most common types of cancer. At least 40% of all cancers worldwide are skin cancers. This cancer is on the rise with a terrible trend. Twenty percent of Americans have the disease, of which more than 36,000 are women and have been diagnosed with melanoma. Therefore, early detection of this cancer can play a significant role incurring this cancer and survive from its dangers. Recently, for reducing the experts' errors, image processing techniques have been employed for these purposes. These techniques can play a complementary role alongside of the experts. Therefore, in the present study, an optimal computer-aided diagnosis system based on deep learning was proposed for early detection of the skin cancer. The idea was to propose an optimized version of Inception convolutional neural network for features extraction from the skin cancer images. The results features were then pruned by the Wildebeest Herd Optimization (WHO) Algorithm as a feature selection technique. Using the WHO algorithm is to select just the useful features and to neglect the irrelevant ones. After designing the method, it was applied to a standard dataset, namely, International Skin Imaging Collaboration (ISIC-2008) dataset with over 13,000 dermoscopic images. The simulation results of the proposed method were compared with Chimp optimization algorithm (ChOA), Biogeography-Based Optimizer (BBO), and Locust Swarm Optimization (LS) for defining the feature selection efficiency. The results indicated that the proposed method provides better effectiveness in terms of accuracy, minimizing the number of extracted features and the speed. The final diagnosis system were also compared with some well-known methods including Dorj's, Linsangan's, Thanh's, Khan's, and Angurana's methods to show its dominance toward the studied methods. According to the results, the suggested method based on the EHO algorithm and Inception CNN provides the best results among all studied methods. However, the results showed the best results for the proposed WHO algorithm, and some other new metaheuristics can be testified to solve the problems like monarch butterfly optimization (MBO), earthworm optimization algorithm (EWA), elephant herding optimization (EHO), moth search (MS) algorithm, Slime mould algorithm (SMA), and Harris hawks optimization (HHO) which are a good motivation for the future work.

## Figures and Tables

**Figure 1:** An overview of Inception network [14].

**Figure 2:** Some samples of the ISIC-2008 dataset [21].

**Figure 3:** The running time of the analyzed algorithms.

**Figure 4:** The simulation results for number of selected features based on the studied comparative algorithms.

**Figure 5:** The simulation results of the suggested method compared with other state-of-the-art methods.

**Table 1:** The parameter setting of the utilized optimization algorithms.

Algorithm	Parameter	Value
ChOA [22]	*r*_1_ and *r*_2_	Random
	*m*	Chaotic

BBO [23]	Habitat modification probability	1
	Immigration probability bounds per gene	[0, 1]
	Step size for numerical integration of probabilities	1
	Max immigration (*I*) and Max emigration (*E*)	1
	Mutation probability	0.005

LS [24]	*F*	0.6
	*L*	1
	*g*	20

WHO [20]	Inertia	0.2
	*P*_Cross_	0.7
	*P*_Mut_	0.15
	Tour_size_	0.7

**Table 2:** Results of feature selection by the optimization algorithms.

Algorithm	Measurement indicator			
	fit_avg_	Std	fit_Best_	fit_worst_
ChOA [22]	0.215	0.009	0.194	0.308
BBO [23]	0.597	0.034	0.351	0.640
LS [24]	0.085	0.009	0.041	0.062
WHO	0.037	0.005	0.039	0.051

**Table 3:** The simulation results of the suggested method compared with other state-of-the-art methods.

Method	Performance metric					
	DS	ACC	SNS	SPC	NPV	PPV
Dorj's [25]	0.91	0.90	0.93	0.91	0.95	0.85
Linsangan's [26]	0.89	0.84	0.19	0.64	0.87	0.69
Thanh's [6]	0.87	0.85	0.87	0.88	0.88	0.81
Khan's [2]	0.88	0.73	0.86	0.63	0.85	0.62
Angurana's [27]	0.91	0.76	0.84	0.79	0.88	0.78
Proposed method	0.94	0.96	0.96	0.95	0.97	0.89

## Data Availability

The data for the dataset can be obtained in https://www.isic-archive.com/.
